The article "Expression of lncRNA-ANRIL before and after Treatment and Its Predictive Value for Short-Term Survival in Patients with Coronary Heart Disease" was retracted in 2024. Reasons: signs of a paper mill; suspected computer-generated content; unreliable results or conclusions; concerns about the data.

# Expression of lncRNA-ANRIL before and after Treatment and Its Predictive Value for Short-Term Survival in Patients with Coronary Heart Disease

**DOI:** 10.1155/2021/5431985

**Published:** 2021-12-03

**Authors:** Jinhui Sun, Shi Qiu

**Affiliations:** Department of Cardiovascular Surgery, The Second Hospital of Shandong University, Jinan 250000, China

## Abstract

This study aimed at observing the expression of lncRNA-ANRIL (ANRIL) before and after treatment and its predictive value for short-term survival in patients with coronary heart disease (CHD). Altogether, 112 patients with CHD admitted to the hospital were enrolled as a study group (SG), which was divided into a pretreatment study group (preSG) and a posttreatment study group (postSG). Further 72 healthy people undergoing physical examinations during the same period were enrolled as a control group (CG). Peripheral blood was collected from the subjects in the three groups, to detect the expression level of serum ANRIL using quantitative reverse transcription PCR (qRT-PCR). A receiver operating characteristic (ROC) curve was plotted to evaluate the diagnostic value of ANRIL for CHD. Kaplan-Meier survival curves were plotted to analyze 3-year survival rates in high- and low-ANRIL expression groups. Cox regression was conducted to analyze independent risk factors affecting the patients. The expression level of serum ANRIL in preSG was significantly lower than those in CG and postSG (*P* < 0.05). According to the ROC curve, the area under the curve (AUC) of serum ANRIL for diagnosing CHD in CG was 0.894 and the optimal cutoff value was 0.639, with the sensitivity of 86.61% and the specificity of 93.67%. According to the survival curves, the 3-year overall survival rate in the high-ANRIL expression group was significantly lower than that in the low-expression group (*P* < 0.05). History of smoking, high total cholesterol (TC), high triglyceride (TG), high homocysteine (Hcy), and ANRIL expression were independent prognostic factors affecting the overall survival time of the patients (*P* < 0.05). ANRIL is poorly expressed in the peripheral blood of patients with CHD. Its detection has good sensitivity and specificity for diagnosing the disease, and its expression may be related to the poor prognosis of the patients.

## 1. Introduction

Coronary heart disease (CHD) is a major cause of patient death in developing countries [1] and a main reason for diseases and disabilities [2, 3]. The shortage of blood and oxygen supply or the occlusion or stenosis of coronary arteries leads to myocardial dysfunction, thus resulting in myocardial infarction, unstable angina pectoris, and heart failure [4–6]. CHD has an increasing incidence with the aging of the population [7] and changing disease conditions. Therefore, it is necessary to explore new biomarkers that are helpful for the better diagnosis of the disease.

Long noncoding RNAs (lncRNAs), as a new type of noncoding RNA, play a vital role in chromatin modification, cell differentiation and proliferation, translation, transcription, and other biological processes [8–10]. According to previous studies, many disordered lncRNAs that are found in various tumors can regulate gene transcription and then play an important role in tumorigenesis and they can also act as tumor suppressor genes or oncogenes [11]. Increasing evidences show that lncRNAs play vital roles in regulating the apoptosis of myocardial cells in myocardial ischemia/reperfusion injury [12–14]. Long non-coding RNA antisense noncoding RNA at the INK4 locus (ANRIL), also known as lncRNA CDKN2B-AS1, is firstly found in patients with hereditary melanoma and neural system tumor. Studies have shown that abnormally expressed ANRIL is observed in various cancers [10, 11]. Besides, the decrease of ANRIL in intestinal mucosa exhibited a relationship to the increase of inflammation, severity, and risk of Crohn's disease [12]. ANRIL gene has been identified as a genetic susceptibility locus related to type 2 diabetes, CHD, intracranial aneurysm, and cancers in genome-wide association studies of common diseases. Importantly, ANRIL is correlated with atherosclerotic cardiovascular disease by genome-wide association studies [13]. What is more, ANRIL is remarkably upregulated in left ventricle biopsies and peripheral blood mononuclear cells of heart failure patients than control subjects [14], implying that ANRIL was probably involved in heart disease regulation [15]. Zhang et al. reported that overexpressing ANRIL can upregulate vascular endothelial growth factors by activating the nuclear factor *κ*B (NF-*κ*B) signaling pathway in rats to promote angiogenesis [16]. Song et al. found that ANRIL plays a protective role in the treatment of patients with aggravated coronary atherosclerosis. It reduces the apoptosis of vascular endothelial cells and the expression of inflammatory cytokines by reducing its own expression, thereby preventing the development and progression of coronary atherosclerosis [17]. However, there are currently few studies on the predictive value of serum ANRIL in the diagnosis of and the therapeutic effect on CHD.

In this study, the expression of serum ANRIL in patients with CHD was examined and its role in the diagnosis and prognosis of the patients was explored.

## 2. Materials and Methods

### 2.1. General Information

A total of 112 patients with CHD admitted to the Department of Cardiology in The Second Hospital of Shandong University from May 2015 to February 2016 were enrolled as the study group (SG), which was divided into a pretreatment study group (preSG) and a posttreatment study group (postSG). These patients met the inclusion criteria stated in our study. The patients in SG consisted of 55 males and 57 females, among whom 51 were <60 years old and 61 were ≥60 years old. Further 72 healthy people undergoing physical examinations during the same period were enrolled as the control group (CG), including 34 males and 45 females, among whom 39 were <60 years old and 40 were ≥60 years old. All participants were informed of this study and signed the informed consent form. Our whole research was approved by the Ethics Committee of The Second Hospital of Shandong University.

### 2.2. Inclusion and Exclusion Criteria

Inclusion criteria were as follows: patients diagnosed with CHD by coronary angiography at admission [18], patients with stable vital signs, patients with complete general information, patients conforming to indications for PCI, patients whose expected survival time ≥ 1 year, male patients aged 60–82 years, and nonpregnant females. Exclusion criteria were as follows: patients with a stress state; patients with arrhythmia or acute myocardial infarction; patients complicated with valvular disease; patients with hyperthyroidism, infectious diseases, or hematopoietic failure; elderly patients with CHD; patients with mental disorders or a family history of mental diseases; patients with severe hepatic and renal dysfunction; patients with chronic obstructive pulmonary disease; patients who transferred to other hospitals halfway; patients who received other hospitals' treatment without authorization; and patients who withdrew from this experiment halfway.

### 2.3. Therapeutic Methods

Patients with CHD were treated with aspirin, angiotensin converting enzyme, receptor blockers, nitrates, and other drugs for lowering lipid. All of them were treated for one month according to the doctor's advice.

### 2.4. Experimental Steps

The serum was collected from the research objects in CG, preSG, and postSG for extracting total RNA using a TRIzol kit (Shanghai Lianshuo Biotechnology Co. Ltd., item no. Invitrogen 15596-026). The concentration and purity of the extracted total RNA were detected with an ultraviolet spectrophotometer (PKUCare Industrial Park Technology Co. Ltd., item no: UV-1100), and its integrity was detected with 1% agarose gel electrophoresis. According to the instruction of the reverse transcription kit (Beijing Protein Innovation Co. Ltd., item no.: BPI01030), the RNA was reversely transcribed into cDNA, which was stored at −80°C for later use. With GAPDH considered as an internal reference, upstream and downstream sequences of ANRIL were 5′-TTATGCTTTGCAGCACACTGG-3′ and 5′-GTTCTGCCACAGCTTTGATCT-3′ and those of GAPDH were 5′-GGGAAACTGTGGCGTGAT-3′ and 5′-GAGTGGGTGTCGCTGTTGA-3′. The reaction was carried out on the real-time fluorescence quantitative PCR instrument (Shanghai Sunshine Biotech Co. Ltd., item no.: qTOWER3G). Conditions for PCR amplification were as follows: predenaturation at 95°C for 30 s, cycling (denaturation at 95°C for 40 min and annealing) for 40 times, standing at 55°C for 1 min, and then extension at 40°C for 5 min. Three independent experiments were carried out to obtain data, and the relative expression of the genes was expressed after calculated by 2^−∆∆*CT*^.

### 2.5. Follow-up

All patients were followed up for 3 years, once every 3 months, up to March 2019. The overall survival time was from the first day after treatment to the last follow-up or patient death.

### 2.6. Statistical Analysis

SPSS17.0 (IBM Corp., Armonk, NY, USA) was used to statistically analyze the data. GraphPad Prism 6 (GraphPad Software, San Diego, USA) was used to plot figures. Measurement data were expressed by mean ± standard deviation (−*x* ± sd), and the comparison of the data between two groups was conducted by independent samples *t*-test. Count data were expressed by the number of cases/percentage [*n*(%)]. A receiver operating characteristic (ROC) curve was plotted to evaluate the diagnostic value of serum ANRIL for diagnosing CHD in CG. Independent prognostic factors for the disease were tested by Cox proportional hazards model. *P* < 0.05 indicated a statistically significant difference.

## 3. Results

### 3.1. Comparison of General Information

There were no significant differences between SG and CG in gender, age, body mass index (BMI), course of disease, place of residence, nationality, educational background, history of smoking, history of drinking, history of diabetes, history of hypertension, types of CHD, and work history (*P* > 0.05). See Table 1.

### 3.2. Relative Expression of Serum ANRIL before Treatment

The expression of serum ANRIL was (0.409 ± 0.12) ng/mL in CG, (0.959 ± 0.16) ng/mL in preSG, and (0.413 ± 0.13) ng/mL in postSG. The expression in preSG was significantly higher than those in CG and postSG (both *P* < 0.05). See Figure 1.

### 3.3. Relationship between Pathological Parameters and Expression of ANRIL

There were significant differences in the relative expression of ANRIL between CHD patients with different ages, history of smoking, history of hypertension, high total cholesterol (TC), high triglyceride (TG), and high homocysteine (Hcy) (*P* < 0.05), not between those with different genders, types of CHD, history of drinking, and history of diabetes (*P* > 0.05). See Table 2.

### 3.4. Diagnostic Value of Serum ANRIL in SG

According to the ROC curve, ANRIL had a better diagnostic value in SG. The area under the curve (AUC) of serum ANRIL for diagnosing CHD in CG was 0.894, and the optimal cutoff value was 0.639, with the sensitivity of 86.61% and the specificity of 93.67%. See Table 3 and Figure 2.

### 3.5. Survival of Patients with CHD

With the median relative expression of serum ANRIL as the critical value, there were 57 cases in the high-ANRIL expression group (<0.639) and 55 cases in the low-ANRIL expression group (≥0.639). The 3-year overall survival rate in the high-expression group was 82.46% (47/57), significantly lower than 94.55% (52/55) in the low-ANRIL expression group (*P* < 0.05). See Figure 3.

The 3-year overall survival rate in the high-ANRIL expression group was significantly lower than that in the low-ANRIL expression group (*P* < 0.05).

### 3.6. Analysis of Prognostic Factors Related to CHD

The univariate analysis was conducted on general and clinicopathological factors. The results showed that gender, types of CHD, history of drinking, and history of diabetes were not prognostic factors affecting the overall survival time of the patients (*P* > 0.05). Different ages, history of smoking, history of hypertension, high TC, high TG, high Hcy, and ANRIL expression may be the prognostic factors (*P* < 0.05). See Table 4. After the significant indicators in the univariate analysis were incorporated into the Cox proportional hazards model, multivariate analysis was conducted through a stepwise regression method. Criteria for variable entry and elimination were 0.05 and 0.1, respectively. The results showed that history of smoking, high TC, high TG, high Hcy, and ANRIL expression were independent prognostic factors affecting the overall survival time (*P* < 0.05). See Table 5.

## 4. Discussion

CHD is a major cause of pathogenesis and patient death in the world [19, 20] and accounts for 2/3 of the death toll from heart disease [21]. The diagnosis and treatment of CHD have been greatly improved in the past decade, but its incidence and mortality have not significantly decreased [22, 23]. At present, the gold standard for diagnosing the disease is coronary angiography, which has a high risk and an expensive cost and cannot assess microcirculation [24]. Therefore, a noninvasive biomarker with satisfactory sensitivity and specificity should be found to diagnose CHD and monitor its disease activity. Accordingly, it is necessary to further explore a new biomarker that can diagnose the disease and predict its condition more effectively.

At present, the pathogenesis of CHD remains unclear but some scholars have reported the abnormal expression of lncRNA as a tumor suppressor gene or oncogene in patients with CHD. According to Wang et al., interferon-y and lncRNA-BANCR play a pivotal role in CHD and they may be used as biomarkers for the screening and prevention of the disease in clinical practice [25]. According to Yin et al., lncRNA-CAS5 acts as an upstream regulator in the mTOR signaling pathway to participate in the progression of CHD and its expression is specially downregulated in patients with the disease, so it can be used as a biomarker for the disease [26]. In our study, the relative expression of serum ANRIL in preSG was significantly higher than those in CG and postSG; ANRIL was closely related to different ages, history of smoking, history of hypertension, high TC, high TG, and high Hcy. These findings indicate that ANRIL may become a potential and analytical marker for CHD in the diagnosis of clinical parameters. According to Samanta and others, hypertension, diabetes, drinking, high TC, and tobacco smoke exposure are additive effects leading to heart disease [27]. According to Li et al., smoking, hyperuricemia, drinking, and BMI are risk factors for the increasing pathogenesis and death risks of CHD in the 55–64 age group [28], which is similar to the results of this study. In our further research, after treatment, the expression level of ANRIL significantly decreased; the AUC of serum ANRIL alone for diagnosing CHD was 0.894, and the optimal cutoff value was 0.639, with the sensitivity of 86.61% and the specificity of 93.67%. These findings suggest that the therapeutic effect on CHD can be predicted by observing changes in the ANRIL expression level. There is currently little research on whether ANRIL affects the therapeutic effect. In our study, patients with high-ANRIL expression had an increasing risk of ineffective treatment. Therefore, observing the expression of ANRIL is helpful to judge the therapeutic effect on patients with CHD. Finally, 112 patients in this study were followed up for 3 years. The overall 3-year survival rate in the high-ANRIL expression group (82.46%) was significantly lower than that in the low-ANRIL expression group (94.55%). According to the univariate analysis of the Cox proportional hazards model, different ages, history of smoking, history of hypertension, high TC, high TG, high Hcy, and ANRIL expression may be prognostic factors affecting the overall survival time. The analysis of the results shows that the high expression of ANRIL promotes the progression of CHD and that history of smoking, high TC, high TG, and high Hcy are the factors affecting the prognosis of patients with CHD. This reveals that ANRIL is a potential factor for judging the prognosis.

This study confirms the value of serum ANRIL for diagnosing CHD and for evaluating the therapeutic effect on the disease, but it still can be improved. Firstly, the relationship between ANRIL and toxic and side effects during treatment should be further addressed. Secondly, the specific regulatory mechanism of ANRIL in the treatment needs to be discussed. Additionally, the influence of ANRIL on tumor formation in mice can be supplemented. Furthermore, the clinical and molecular mechanism research on rare cases of CHD should be studied.

To sum up, ANRIL is highly expressed in the serum of patients with CHD and it can be used as an effective biomarker for evaluating the therapeutic effect on the disease and the 3-year overall survival rate of the patients.

## Figures and Tables

**Figure 1:** Relative expression of serum ANRIL before treatment. The expression of serum ANRIL in preSG was significantly higher than that in CG and postSG (*P* < 0.05). ^∗∗∗^*P* < 0.05.

**Figure 2:** ROC curve of serum ANRIL for diagnosing coronary heart disease.

**Figure 3:** 3-year survival of patients with coronary heart disease.

**Table 1:** Comparison of general information [*n*(%)] (−*x* ± sd).

Categories	SG (*n* = 112)	CG (*n* = 79)	*t*/*χ*^2^ value	*P* value
Gender			0.687	0.408
Male	55 (49.11)	34 (43.04)		
Female	57 (50.89)	45 (56.96)		
Age (years)			0.273	0.601
<60	51 (45.54)	39 (49.37)		
≥60	61 (54.46)	40 (50.63)		
BMI (kg/m^2^)			1.521	0.129
	23.4 ± 3.7	22.6 ± 3.4		
Place of residence			0.933	0.334
City	66 (58.93)	52 (65.82)		
Countryside	46 (41.07)	27 (34.18)		
Nationality			0.035	0.851
Han	58 (51.79)	42 (53.16)		
National minorities	54 (48.21)	37 (46.84)		
Educational history			0.984	0.321
≥senior high school	43 (38.39)	36 (45.57)		
<senior high school	69 (61.61)	43 (54.43)		
History of smoking			0.525	0.469
Yes	57 (50.89)	36 (45.57)		
No	55 (49.11)	43 (54.43)		
History of drinking			0.078	0.781
Yes	53 (47.32)	39 (49.37)		
No	59 (52.68)	40 (50.63)		
History of diabetes			1.862	0.172
Yes	58 (51.79)	33 (41.77)		
No	54 (48.21)	46 (58.23)		
History of hypertension			2.889	0.089
Yes	65 (58.04)	36 (45.57)		
No	47 (41.96)	43 (54.43)		
Work history			0.189	0.663
Yes	33 (29.46)	21 (26.58)		
No	79 (70.54)	58 (73.42)		

BMI: body mass index.

**Table 2:** Relationship between clinicopathological parameters and relative expression of ANRIL in peripheral blood (−*x* ± sd).

Pathological parameters	n	Relative expression of ANRIL	*t*/*F*	*P*
Gender			0.146	0.884
Male	55	0.957 ± 0.15		
Female	57	0.961 ± 0.14		
Age (years)			2.030	0.045
<60	51	0.930 ± 0.13		
≥60	61	0.978 ± 0.12		
Types of CHD			0.001	0.993
Angina pectoris	35	0.958 ± 0.15		
Remote myocardial infarction	33	0.962 ± 0.14		
Acute myocardial infarction	44	0.959 ± 0.14		
History of smoking			0.401	0.689
Yes	57	0.952 ± 0.15		
No	55	0.963 ± 0.14		
History of drinking			0.188	0.852
Yes	53	0.962 ± 0.13		
No	59	0.957 ± 0.15		
History of diabetes			0.127	0.899
Yes	58	0.961 ± 0.12		
No	54	0.958 ± 0.13		
History of hypertension			2.059	0.042
Yes	65	0.984 ± 0.12		
No	47	0.935 ± 0.13		
TC (mmol/L)			2.039	0.044
≥4.34	63	0.987 ± 0.15		
<4.34	49	0.932 ± 0.13		
TG (mmol/L)			1.995	0.049
≤1.93	68	0.941 ± 0.11		
>1.93	44	0.985 ± 0.12		
Hcy (*μ*mol/L)			2.049	0.043
≤16.8	67	0.939 ± 0.12		
>16.8	45	0.988 ± 0.13		

CHD: coronary heart disease (CHD); TC: total cholesterol; TG: triglyceride; Hcy: high homocysteine.

**Table 3:** Diagnostic value of serum ANRIL in SG.

Diagnostic index	AUC	95% CI	Standard error	Cutoff value	Sensitivity (%)	Specificity (%)
ANRIL	0.894	0.841~0.947	0.027	0.639	86.61	93.67

**Table 4:** Univariate analysis of prognostic factors for patients with CHD.

Groups	Number of investigation (cases)	Number of 3-year survival (cases)	*χ* ^2^	*P*
Gender			2.068	0.150
Male	55	33		
Female	57	52		
Age (years)			0.013	0.908
<60	51	38		
≥60	61	47		
Types of CHD			0.565	0.754
Angina pectoris	35	29		
Remote myocardial infarction	33	21		
Acute myocardial infarction	44	35		
History of smoking			4.439	0.035
Yes	57	56		
No	55	29		
History of drinking			0.016	0.899
Yes	53	41		
No	59	44		
History of diabetes			0.028	0.868
Yes	58	43		
No	54	42		
History of hypertension			0.148	0.700
Yes	65	47		
No	47	38		
TC (mmol/L)			4.987	0.026
≥4.34	63	61		
<4.34	49	24		
TG (mmol/L)			5.470	0.019
≤1.93	68	65		
>1.93	44	20		
Hcy (*μ*mol/L)			4.401	0.036
≤16.8	67	63		
>16.8	45	22		
ANRIL expression			3.987	0.046
Low expression	55	52		
High expression	57	47		

CHD: coronary heart disease (CHD); TC: total cholesterol; TG: triglyceride; Hcy: high homocysteine.

**Table 5:** Multivariate analysis of prognostic factors for patients with CHD.

Projects	Multivariate	
	HR (95% CI)	*P*
History of smoking	1.46 (1.04~2.67)	0.035
TC	1.77 (1.13~2.74)	0.012
TG	1.66 (1.12~2.87)	<0.001
Hcy	1.79 (1.21~3.10)	<0.001
ANRIL low expression	2.32 (1.46~3.69)	<0.001

CHD: coronary heart disease (CHD); TC: total cholesterol; TG: triglyceride; Hcy: high homocysteine.

## Data Availability

The datasets used and/or analyzed during the present study are available from the corresponding author on reasonable request.
